# Effects of Bevacizumab Combined with Chemotherapy on CT, CyFRA21-1, and ProGRP and Prognosis of Lung Cancer Patients under Nursing Intervention

**DOI:** 10.1155/2022/9422902

**Published:** 2022-07-14

**Authors:** Chao Xi, Hong Jiang, Yinling Xue, Yongmei Lv, Chao Wang

**Affiliations:** ^1^Department of Thoracic Surgery, Zhangqiu District People's Hospital, Jinan 250200, China; ^2^Department of Imaging, Yantai Yuhuangding Hospital Affiliated to Qingdao University, Yantai 264000, China; ^3^Department of Urology Surgery, Qingdao Hospital of Traditional Chinese Medicine, Hiser Medical Group of Qingdao, Qingdao 266033, China; ^4^Department of Pharmacy, Zhangqiu District People's Hospital, Jinan 250200, China; ^5^Department of Pharmacy, Qingdao Hospital of Traditional Chinese Medicine, Hiser Medical Group of Qingdao, Qingdao 266033, China

## Abstract

**Objective:**

Molecular targeted drug therapy and chemotherapy are the main treatments for advanced non-small-cell lung cancer, and the combination of both has advantages in prolonging patients' progression-free survival and overall survival. This study investigated the effects of bevacizumab combined with chemotherapy under nursing intervention on CT, cytokeratin 19 fragment antigen 21-1 (CYFRA21-1), and gastrin-releasing peptide precursor (ProGRP) and prognosis of lung cancer patients.

**Methods:**

102 patients with non-small-cell lung cancer admitted to our hospital from January 2018 to May 2019 were divided into observation group and control group, with 51 cases each. The control group was treated with basic chemotherapy, and the observation group was treated with bevacizumab in combination with the control group, and both groups used nursing interventions. The clinical effects, CYFRA21-1 and ProGRP levels, baseline data, CT parameters, 24-month cumulative survival, and the effects of CYFRA21-1 and ProGRP on long-term survival and lung function were compared.

**Results:**

The disease control rate of the observation group was 94.12%, which was significantly higher than that of the control group (76.47%); after 7 d, 30 d, 60 d, and 90 d of treatment, the levels of CYFRA21-1 and ProGRP were statistically downregulated. The difference in lymph node metastasis, lesion diameter, plain Eff-Z, venous stage, and arterial stage normalized iodine concentrations (NIC) was statistically significant; the survival rate at 24 months in the observation group was 74.51% (38/51); the cumulative survival rate at 24 months in the control group was 52.94% (27/51), and the difference was statistically significant (*X*^2^ = 4.980, *P* = 0.026). The cumulative survival rate at 24 months was significantly lower in patients with high expression of CYFRA21-1 and ProGRP compared with those with low expression of CYFRA21-1 and ProGRP. After treatment, in the observation group, the forceful spirometry (FVC), forceful expiratory volume in one second (FEV1), and FEV1/FVC levels were significantly different from those before treatment and were significantly different from those in the control group.

**Conclusion:**

Bevacizumab in combination with standard chemotherapy regimens with nursing interventions could benefit patients with advanced non-small-cell lung cancer and had a good prospect of application.

## 1. Introduction

Lung cancer is known as primary bronchial lung cancer, and the incidence rate and death rate of lung cancer in China have been increasing year by year in recent years. Lung cancer is divided into small cell lung cancer (SCLC) and non-small-cell lung cancer (NSCLC), of which NSCLC accounts for more than 80% of all lung cancers [1–3]. There are no typical manifestations in the early stage of lung cancer, and its clinical symptoms are easily confused with other benign lung and respiratory tract lesions, and local spread or distant metastasis has occurred when it progresses to the middle and late stages [4].

Currently, clinical treatment of lung cancer is mainly based on radiotherapy and chemotherapy, which are administered intravenously to induce apoptosis of tumor foci in order to alleviate clinical symptoms. However, long-term clinical studies have found that the use of chemotherapy alone in patients with non-small-cell carcinoma has certain limitations, and the prognosis is not ideal [5–7]. With the continuous development of tumor treatment technology, molecular targeted drug therapy has gradually become the main mode of lung cancer treatment [8, 9]. It has been confirmed by clinical practice that targeted therapy can effectively inhibit tumor cell proliferation, which is of great significance in the treatment of lung cancer [9, 10]. Bevacizumab is the first angiogenesis inhibitor that has been shown to prolong the survival of NSCLC patients in combination with chemotherapy [11]. Akamatsu et al. conducted the first phase III clinical study for Chinese NSCLC patients, and the experimental results showed that the median PFS and OS of paclitaxel + carboplatin combined with bevacizumab were 9.2 and 24.3 months, confirming that bevacizumab combined with chemotherapy could benefit Chinese NSCLC patients [12].

However, while molecularly targeted drugs inhibit tumor cell proliferation and growth in lung cancer patients, they also bring certain risks of adverse effects, causing heavy psychological pressure on patients and leading to negative emotions such as anxiety and depression, which seriously reduce patients' quality of life [13]. This places higher demands on lung cancer nursing, and preventive nursing interventions are a means of emphasizing the safety of the treatment, helping to reduce the burden of multiple symptoms at the physical and psychological levels during treatment, and improving patients' treatment compliance and quality of life [14]. Studies have pointed out that CT is the most commonly used tool for efficacy assessment and is an anatomical imaging technique with good reproducibility, reflecting the patient's condition and predicting the risk of poor prognosis [15]. Cytokeratin 19 fragment antigen 21-1 (CYFRA21-1) levels correlate with tumor load and metastasis in intermediate to advanced NSCLC and can be used as an adjunctive assessment indicator of treatment response and prognosis [16]. Gastrin-releasing peptide precursor (ProGRP) is a new hormonal tumor marker isolated from gastric tissues and widely distributed in gastric nerve fibers and pulmonary neuroendocrine tissues, which is widely used in the diagnosis and monitoring of lung cancer due to its long half-life [17].

In this study, we investigated the clinical efficacy and the effects on CT, CYFRA21-1 level, ProGRP level, and prognosis of 102 lung cancer patients treated with bevacizumab in combination with chemotherapy under preventive care intervention.

## 2. Materials and Methods

### 2.1. General Information

The medical records of lung cancer patients admitted to our hospital from January 2018 to May 2019 were collected. Inclusion criteria are as follows: (i) non-small-cell lung cancer diagnosed by surgical pathology or fiberoptic bronchoscopy biopsy, (ii) no history of radiotherapy, (iii) expected survival time of more than half a year, and (iv) complete clinical data. Exclusion criteria are as follows: (1) patients with contraindications to CT examination or contrast allergy; (2) patients within 14 days after major surgery or trauma; (3) patients in the acute phase of infectious diseases, acute exacerbation of various chronic diseases, and acute phase of adverse events in the cardiovascular and cerebrovascular systems; (4) patients with other lung diseases such as pulmonary vasculopathy, pulmonary encapsulation, tuberculosis, or congenital anatomical abnormalities of the lung or respiratory tract; and (5) the presence of severe psychiatric disorders, cognitive impairment, and communication disorders. A total of 102 lung cancer patients were included in this study and divided into an observation group and a control group with 51 cases each. In the control group, there were 29 males and 22 females, aged 51-68 years, with a mean of 57.63 ± 5.39 years. In the observation group, there were 32 males and 19 females, aged 50-70 years, with an average of 57.41 ± 5.98 years. The differences in gender and age between the two groups were not statistically significant (*P* > 0.05) and were comparable. The study was approved by the hospital ethics committee, and all patients gave their informed consent and signed the informed consent form.

### 2.2. Treatment Method

The control group was treated with a TC chemotherapy regimen: 250 mL of glucose solution mixed with 175 mg/m^2^ paclitaxel (Harbin Labotong Pharmaceutical Co., Ltd., National Drug Administration H20067522, specification: 5 mL: 30 mg) was given intravenously on day 1; on the second day, 250 mL of glucose solution was mixed with 300-400 mg/m^2^ carboplatin (Zhejiang Haisheng Pharmaceutical Co., Ltd., National Drug Administration H20044177, specification: 100 mg) and then administered intravenously. 21 d was a course of treatment, and there were 3 courses of treatment, with an interval of 1 week between each course.

In the observation group, bevacizumab targeting therapy was given in combination with the TC chemotherapy regimen. The TC chemotherapy regimen was the same as that of the control group. 7.5 mg/m^2^ bevacizumab injection was given intravenously on day 1 of chemotherapy. 21 d was a course of treatment, once for each course of treatment, and the efficacy was evaluated after 3 courses of treatment.

### 2.3. Nursing Method

Nursing interventions were implemented [18].

1. *Complication Interventions*. Pay attention to the cleanliness and moistening of the patient's radiated skin, avoid direct sunlight stimulation of the irradiated patient's skin, and try to choose clothing made of more comfortable fabrics to avoid damage to the patient's organism skin due to friction. Pay attention to the patient's posture after eating and drinking, and forbid lying down to prevent food reflux, residue, and other foreign bodies, thus preventing esophagitis. Advise the patient to drink plenty of normal temperature water and to choose the appropriate nebulization input to ensure the smooth flow of the airway
2. *Lifestyle Interventions*. Observe and count the daily dietary status of the patient and develop a set of targeted individualized diet plans to ensure the daily intake of vitamins, proteins, and other nutrients. Do not consume spicy and stimulating foods, and follow the principle of small and frequent meals. The decline of the patient's physical quality was associated with the level of care, which may lead to negative phenomena such as irritability and anxiety, so the medical staff should communicate with the patient more often to increase the patient's compliance with treatment and to build up their confidence in overcoming the disease. A certain scale of patient conversation could be carried out to further enhance the patient's treatment initiative
3. *Pain Intervention*. Patients were instructed to carry out healthier physical rehabilitation exercises and targeted interventions such as distraction methods, and watching children's programs and videos were carried out for patients with different pain levels
4. *Psychological Care*. Strengthen communication with patients and help them to adjust their psychological state, and invite patients with successful treatment cases to “present themselves” to enhance their confidence in the treatment and relieve their negative emotions. Patiently explain the role of radiotherapy and the occurrence of gastrointestinal adverse effects as a normal phenomenon to increase treatment confidence

### 2.4. CT Scanning Methods

GE gem energy spectrum CT (Discovery CT750 HD) was used for chest plain scan and two-phase enhanced scan. The scan parameters were as follows: tube voltage was switched between high and low energy (80 kVp and 140 kVp) instantaneously (0.5 ms), automatic milliamp, pitch 1.375 : 1, layer spacing 5.0, layer thickness 5.0 mm, matrix 512 × 512, collimation 64 × 0.625 mm, and frame rotation time 0. 6 s. The scan area included the lung tip to the rib diaphragm angle. After plain scanning, nonionic contrast agent iohexol was injected through the median cubital vein for 1.6 mL·kg^−1^, time ≤ 30 s, and the CT value of the thoracic aorta was monitored. After reaching the threshold value of 150 HU, the scanning was delayed for 5.7 s, and the venous phase images were delayed for 30 s after obtaining arterial phase images. The images were uploaded to the workstation and reviewed by 2 attending physicians. The solid component of the lesion was selected as the region of interest (ROI), and the ROI of each phase was measured once at each of the three adjacent levels, with consistent size, morphology, and location, and the average value was obtained. The effective atomic number (Eff-Z) was recorded, and the normalized iodine concentrations (NIC) were calculated as NIC = iodine content in the ROI of the lesion/aortic iodine content.

### 2.5. Observation Index

1. Compare the clinical efficacy of the two groups after 3 courses of treatment, in which complete remission (CR): CT scan showed no target tumor, no cavity, pulmonary atelectasis, etc.; partial remission (PR): CT scan showed incomplete cavity of the target tumor, containing liquid or solid components, showing contrast enhancement, part of the target tumor had fibrosis, containing solid components, with enhancement; stable disease (SD): CT scan showed part of the target tumor as a solid nodule with no significant change in volume and reinforcing features; disease progression (PD): CT scan showed newly scattered, nodular, irregular eccentric reinforcement around the treated out tumor again. Total effective rate = number of (CR + PR) cases/total number of cases × 100%
2. The levels of CYFRA21-1 and ProGRP were compared between the two groups before treatment and after 7, 30, 60, and 90 d of treatment. 5 mL of fasting venous blood was collected from all patients before treatment and left for 20 min in a sterile and light-proof room at 20~26°C, placed in a centrifuge, centrifuged at 3500 r/min for 10 min with a 10 cm radius, and stored the serum in a refrigerator at -20°C for examination. ProGRP level was detected by enzyme-linked immunoadsordent assay (ELISA), and CYFRA21-1 level was detected by electrochemiluminescence assay
3. The survival time of patients was recorded by telephone call back every three months after the end of 3 courses of treatment or when the patients were reexamined
4. Compare the lung function levels of the two groups before and after 3 courses of treatment, and test their forceful spirometry (FVC) and forceful expiratory volume in one second (FEV1) levels

### 2.6. Statistical Analysis

The SPSS 21.0 statistical software was used to analyze the data, and the measurement data and count data were expressed as $\overset{¯}{x}\pm s$ and %, respectively, and *t* and *χ*^2^ tests were used to compare between two groups. Survival curves were plotted using GraphPad Prism 5 to test the survival of NSCLC patients. The difference was statistically significant at *P* < 0.05.

## 3. Results

### 3.1. Comparison of Clinical Efficacy between the Two Groups

The disease control rate of the observation group was 94.12%, which was significantly higher than that of the control group (76.47%), and the difference was statistically significant (*P* < 0.05) (Table 1).

### 3.2. Comparison of CYFRA21-1 and ProGRP Levels between the Two Groups

After 7 d, 30 d, 60 d, and 90 d of treatment, CYFRA21-1 and ProGRP levels in both groups were gradually adjusted downward, and the differences in CYFRA21-1 and ProGRP levels between the two groups compared with those before treatment were statistically significant (*P* < 0.05), and the levels of CYFRA21-1 and ProGRP in the observation group were significantly lower than those in the control group (*P* < 0.05) (Figure 1).

### 3.3. The Baseline Data and CT Parameters Were Compared

There was no statistically significant difference in the comparison of gender, age, clinical stage, histological staging, degree of differentiation, smoking history, and drinking history (*P* > 0.05); the difference was statistically significant in the comparison of lymph node metastasis, lesion diameter, plain Eff-Z, venous stage, and arterial stage NIC (*P* < 0.05) (Table 2).

### 3.4. The Survival Time of the Two Groups Was Compared

The cumulative survival rate at 24 months in the observation group was 74.51% (38/51); the cumulative survival rate at 24 months in the control group was 52.94% (27/51) (*X*^2^ = 4.980, *P* = 0.026) (Figure 2).

### 3.5. Effect of High and Low Expressions of CYFRA21-1 and ProGRP on Long-Term Survival

The 24-month cumulative survival rate of patients with high CYFRA21-1 and ProGRP expression was significantly lower than that of patients with low CYFRA21-1 and ProGRP expressions (Figure 3).

### 3.6. Comparison of Pulmonary Function

After treatment, the FVC and FEV1 levels in the observation group were 2.55 ± 0.63 L and 2.00 ± 0.46 L, respectively, and the FVC and FEV1 levels in the control group were 2.15 ± 0.61 L and 1.56 ± 0.43 L, respectively. The differences between groups and within groups were statistically significant (both *P* < 0.05). After treatment, the difference in FEV1/FVC between the two groups was statistically significant (both *P* < 0.05) (Figure 4).

## 4. Discussion

Lung cancer is a common respiratory malignancy in clinical practice and has a high incidence and morbidity and mortality rate in China. Some data show [19] that the incidence of non-small-cell carcinoma accounts for about 80% of lung cancer. In the early stage, there are mostly no typical symptoms, mainly manifesting as chest tightness, chest pain, cough, hoarseness, fever, and shoulder pain, which are easily confused with other benign lung diseases, leading to the progression of the disease to the middle and late stages when most patients are diagnosed, and the best time for surgery is missed. Chemotherapy can improve patients' clinical symptoms to a certain extent, but after clinical practice, it is found that single chemotherapy can cause many adverse reactions, which can seriously affect patients' subsequent treatment and daily life and cannot better control the development of tumor [20]. Molecular targeted drug therapy has a wide range of applications and can provide good antitumor support for lung cancer patients in different pathological stages. Moreover, it is easy to operate and highly accepted by patients. However, the long-term use of molecularly targeted drugs during the implementation of targeted therapy for lung cancer patients can easily lead to adverse reactions related to skin reactions mainly [21]. The formation of such problems not only aggravates the painful experience of lung cancer patients but also tends to cause the interruption of targeted therapy. As an important complement to antitumor therapy, the role of nursing care in supporting targeted therapy for lung cancer patients directly affects the recovery status of lung cancer patients. Therefore, it is necessary to select appropriate methods to construct nursing programs for lung cancer targeted therapy patients. In targeted lung cancer therapy, this method uses measures such as missionary intervention, psychological protection intervention, and pain care to improve the risk of adverse reaction formation of targeted therapy, alleviate the severity of adverse reactions of lung cancer patients, and provide the necessary support for targeted antitumor therapy of lung cancer patients.

Bevacizumab, as a targeted drug [22], has the advantages of long half-life, human origin, and high selectivity, which can inhibit the development of tumor cells and play the role of inhibiting tumor cell growth and promoting apoptosis. The results of this study showed that the disease control rates in the observation group were all significantly higher than those in the control group (*P* < 0.05); after treatment, the differences in FVC, FEV1, and FEV1/FVC levels in the observation group were statistically significant compared with those in the control group (*P* < 0.05). It was suggested that bevacizumab combined with chemotherapy regimens and nursing interventions were effective in improving treatment outcomes and lung function in patients with non-small-cell lung cancer. The analysis suggested that bevacizumab initiated complement- and antibody-mediated toxic effects, using the body's immune mechanisms to act as a lethal agent against tumor cells. Combined with chemotherapy and nursing intervention regimens, treatment not only alleviated toxic effects but also increased drug tolerance, which in turn improved treatment outcomes and lung function in patients with non-small-cell lung cancer. CT is a medical imaging method widely used in recent years for the diagnosis of lung cancer. CT can detect overlapping and micronodules and can determine the specific nature of nodules and has a high sensitivity for the diagnosis of independent nodules in the lung [23]. Plain scan Eff-Z, venous phase, and arterial phase NIC can be used to identify the nature of the lesion. Low of the three can reflect the tumor growth and invasive ability, the neovascularization cannot meet the tumor blood supply-demand, and there are more mucus and necrotic components inside the tumor, and microhemorrhage occurs, and the lesion shows insufficient blood supply, which further reflects the high malignancy of the tumor and the high risk of poor prognosis of the patient. ProGRP is a gastrointestinal hormone [24], mostly found in many neuroendocrine tumors [25], which has high sensitivity and specificity for SCLC and is an important serum marker for the diagnosis of SCLC. CYFRA21-1 is a cytokeratin [26] that shows high expression in patients with nonsquamous non-small-cell lung cancer, and the more severe the lesion, the higher the expression level. The results of this study showed that bevacizumab combined with chemotherapy and nursing intervention could effectively reduce the levels of tumor markers CYFRA21-1 and ProGRP in patients with non-small-cell lung cancer. The analysis suggested that bevacizumab inhibited VEGF activity during treatment by binding specifically to VEGF, blocking the nutrient supply to the tumor cell microenvironment, and thus controlling or delaying the formation and proliferation of abnormal neovascularization. In addition, the blocking effect of VEGF to inhibit cell progression also promoted the development of chemotherapeutic drug sensitivity in cancer cells, allowing them to initiate antibody- and complement-mediated toxic effects that used immune mechanisms to destroy cancer cells, thereby reducing or stabilizing serum CYFRA21-1 and ProGRP levels. When bevacizumab was used in combination with a chemotherapy regimen, it could reduce the interstitial pressure in the tumor, enhance the permeability of chemotherapy drugs, improve the effectiveness of treatment, and have a good chemotherapy sensitization effect, which could not only enhance the drug tolerance but also reduce the degree of toxic side effects and symptoms, so that the physical function and health condition of patients could be greatly enhanced, and thus improve the survival time of patients after treatment. Therefore, this study also found that bevacizumab not only improved the treatment effect but also had a good prognosis and a high safety profile.

## 5. Conclusion

In conclusion, bevacizumab targeted therapy combined with chemotherapy and nursing intervention could improve the clinical outcome and lung function of patients with non-small-cell lung cancer and reduce serum CYFRA21-1 and ProGRP levels while improving the survival time of patients with good prognosis and high safety, which was worthy of clinical reference.

## Figures and Tables

**Figure 1:** Comparison of cyFRA21-1 and ProGRP levels between the two groups. (a) After 7 d, 30 d, 60 d, and 90 d of treatment, CyFRA21-1 levels were gradually decreased. (b) After 7 d, 30 d, 60 d, and 90 d, ProGRP levels in both groups were gradually downregulated.

**Figure 2:** Comparison of survival time between the two groups.

**Figure 3:** Influence of high and low expressions of CyFRA21-1 and ProGRP on long-term survival.

**Figure 4:** Comparison of lung function between the two groups. (a) Comparison of FEV1 level before and after treatment in the observation group. (b) Comparison of FEV1 levels in the control group before and after treatment. (c) Comparison of FVC levels in the observation group before and after treatment. (d) Comparison of FVC levels in the control group before and after treatment. (e) Comparison of FEV1/FVC levels in the experimental group before and after treatment. (f) Comparison of FEV1/FVC levels in the control group before and after treatment.

**Table 1:** Comparison of clinical efficacy between the two groups (*n* (%)).

Group	*n*	CR	PR	SD	PD	Disease control rate
Observation group	51	26 (50.98)	13 (25.49)	9 (17.65)	3 (5.88)	48 (94.12)
Control group	51	18 (35.29)	9 (17.65)	12 (23.53)	12 (23.53)	39 (76.47)
*X* ^2^						8.010
*P*						0.046

**Table 2:** Comparison of baseline data and CT parameters between the two groups.

Baseline data and CT parameters		Observation group (*n* = 51)	Control group (*n* = 51)	*X* ^2^/*t*	*P*
Gender	Male	32	29	*X* ^2^ = 0.367	0.545
	Female	19	22		
Age (years)	≥55	28	30	*X* ^2^ = 0.160	0.689
	<55	23	21		
Clinical stages	III stage	18	21	*X* ^2^ = 0.374	0.541
	IV stage	33	30		
Histological staging	Adenocarcinoma	26	28	*X* ^2^ = 0.171	0.918
	Squamous carcinoma	17	16		
	Adenosquamous carcinoma	8	7		
Degree of differentiation	Well differentiated	29	28	*X* ^2^ = 0.318	0.853
	Moderately differentiated	19	21		
	Poorly differentiated	3	2		
Smoking history	Yes	32	36	*X* ^2^ = 0.706	0.401
	No	19	15		
Drinking history	Yes	41	42	*X* ^2^ = 0.065	0.799
	No	10	9		
Lymph node metastasis	Yes	4	14	*X* ^2^ = 6.746	0.009
	No	47	37		
Lesion diameter/cm	≥3.5	6	15	*X* ^2^ = 4.411	0.036
	<3.5	45	38		
Plain Eff-Z		7.91 ± 0.46	7.53 ± 0.43	*t* = 4.385	<0.001
Venous stage NIC/mg·cm^−3^		0.41 ± 0.11	0.300 ± 0.08	*t* = 5.696	<0.001
Arterial stage NIC/mg·cm ^−3^		0.16 ± 0.05	0.09 ± 0.02	*t* = 8.609	<0.001

## Data Availability

The data used to support the findings of this study are available from the corresponding author upon request.
